The article "Diverse Fate of an Enigmatic Structure: 200 Years of Meckel’s Cartilage" was published in 2020. Journal: Front Cell Dev Biol.

# Diverse Fate of an Enigmatic Structure: 200 Years of Meckel’s Cartilage

**DOI:** 10.3389/fcell.2020.00821

**Published:** 2020-08-28

**Authors:** Eva Svandova, Neal Anthwal, Abigail S. Tucker, Eva Matalova

**Affiliations:** ^1^Institute of Animal Physiology and Genetics, Academy of Sciences, Brno, Czechia; ^2^Centre for Craniofacial and Regenerative Biology, King’s College London, Guy’s Hospital, London, United Kingdom; ^3^Department of Physiology, University of Veterinary and Pharmaceutical Sciences, Brno, Czechia

**Keywords:** jaw development, craniofacial, mammal evolution, congenital birth defects, chondrogenesis

## Abstract

Meckel’s cartilage was first described by the German anatomist Johann Friedrich Meckel the Younger in 1820 from his analysis of human embryos. Two hundred years after its discovery this paper follows the development and largely transient nature of the mammalian Meckel’s cartilage, and its role in jaw development. Meckel’s cartilage acts as a jaw support during early development, and a template for the later forming jaw bones. In mammals, its anterior domain links the two arms of the dentary together at the symphysis while the posterior domain ossifies to form two of the three ear ossicles of the middle ear. In between, Meckel’s cartilage transforms to a ligament or disappears, subsumed by the growing dentary bone. Several human syndromes have been linked, directly or indirectly, to abnormal Meckel’s cartilage formation. Herein, the evolution, development and fate of the cartilage and its impact on jaw development is mapped. The review focuses on developmental and cellular processes that shed light on the mechanisms behind the different fates of this cartilage, examining the control of Meckel’s cartilage patterning, initiation and maturation. Importantly, human disorders and mouse models with disrupted Meckel’s cartilage development are highlighted, in order to understand how changes in this cartilage impact on later development of the dentary and the craniofacial complex as a whole. Finally, the relative roles of tissue interactions, apoptosis, autophagy, macrophages and clast cells in the removal process are discussed. Meckel’s cartilage is a unique and enigmatic structure, the development and function of which is starting to be understood but many interesting questions still remain.

## Introduction

The developing face is created by a fusion of a number of facial processes, with the lower jaw created by cells largely from the first pharyngeal arch. The structure of the face is first outlined by the cartilaginous chondrocranium, with a single cartilage defining the lower jaw, known as Meckel’s cartilage (MC). MC was first described in mammals by the German anatomist Johann Friedrich Meckel the Younger in the Handbuch der menschlichen Anatomie (Meckel, 1820), 200 years ago. Here Meckel described the relationship between a cartilage rod that ran along the jaw and the forming malleus, and compared this rod to similar structures previously described in fish, amphibians and birds (Meckel, 1820). The cartilage was later named Meckel’s cartilage by his followers (Amano et al., 2010). During development, MC begins life as two rods of cartilage, which meet in the midline to form a V-structure outlining the forming lower jaw (Figures 1A,B). After the first wave of chondrogenesis, the membranous bones form around the cartilaginous templates to create the dermatocranium, with secondary cartilages capping the bones at key points of articulation and mechanical force (Depew et al., 2002). Meckel’s cartilage forms the lower jaw strut in all jawed vertebrates during embryonic development, and as such plays a key conserved role in vertebrate jaw development and evolution (Anthwal et al., 2013). In mammals, the main body of Meckel’s cartilage is largely transient but acts as a template for later formation of the bones of the lower jaw, with defects leading to anomalies in the pattern and size of the jaw in mouse mutants and in human embryos (Bhaskar et al., 1953; Amano et al., 2010). In addition to its role as a jaw support, MC also forms two of the three mammalian middle ear bones (malleus and incus), which sit in the middle ear cavity and, along with the stapes, form a chain of ossicles to transfer sound from the outer to the inner ear. MC function therefore spans both roles in feeding and hearing.

The article "Diverse Fate of an Enigmatic Structure: 200 Years of Meckel’s Cartilage" was published in 2020. Journal: Front Cell Dev Biol.

**FIGURE 1:** Position of Meckel’s cartilage in the mandible and its different developmental fates. Original schematic showing a frontal section of the intermediate part of the murine mandible **(A)**, longitudinal section of the murine mandible **(B)**, sagittal section of the murine mandible **(C)**. Molar/incisor (green), mandibular bone (grey), Meckel’s cartilage (yellow).

In this review the development of the mammalian MC is followed from initiation to final function, highlighting the molecular mechanisms involved in its creation, remodelling and loss, as documented in the research literature. In particular we aim to put into context the recent discoveries in MC development since the last review on this subject (Amano et al., 2010), and highlight the gaps that call for further study of this important cartilage. Over the last ten years, the use of conditional transgenic mice has revealed many of the molecular aspects of MC, providing an understanding of the spatial and temporal dynamics of lower jaw development, and highlighting roles for processes such as autophagy. Likewise the recent use of mammalian models outside mice has shed light on the level of conservation of many of these processes, and the relevance to human development and congenital defects. The fate of different parts of MC in mammals, however, is still unclear, along with the stimuli, both mechanical or molecular, that trigger the changes during ossification, resorption and transformation.

The article "Diverse Fate of an Enigmatic Structure: 200 Years of Meckel’s Cartilage" was published in 2020. Journal: Front Cell Dev Biol.

## Meckel’s Cartilage: A Key Feature of Jawed Vertebrates

Meckel’s cartilage is present in all jawed vertebrates (gnathostomes), and has been hypothesised to have evolved from the ventral gill support structures of the first pharyngeal arch of jawless fish (agnathians) (Mallat, 2008). However, MC may alternatively have formed *de novo* from first arch derived crest in jawed vertebrates. The specialisation of the first arch was a key process in the evolution of jaws, and as such the specification of MC was necessary for the emergence of jawed vertebrates (see Donoghue et al., 2006; Brazeau and Friedman, 2015; Maier and Ruf, 2016; Miyashita, 2016; DeLaurier, 2019; Woronowicz and Schneider, 2019 for further information on the history and evolutionary origins of MC and the jaw). Among non-mammalian jawed vertebrates, MC remains largely cartilaginous in the adult, and acts as a permanent scaffold around which the membranous bones of the mandible are positioned. In these non-mammalian jawed vertebrates, the proximal portion of MC ossifies to form the bones that articulate the upper and lower jaw, with the articular and the quadrate part of the palatoquadrate forming from the same type II collagen expressing condensation in the chick (Wilson and Tucker, 2004). The joint marker *Bapx1* turns on between the quadrate and articular in the chick, creating distinct alcian blue expressing skeletal elements (Wilson and Tucker, 2004).

Uniquely in extant mammals, instead of forming the bones of the jaw joint, the proximal portion of MC ossifies and forms the malleus and incus, two bones of the mammalian three ossicle middle ear (Figure 1C). The malleus is homologous to the articular, while the incus is homologous to the quadrate, with a *Bapx1*-expressing joint forming between the two (Tucker et al., 2004). The incus, malleus and MC are initially united as a single type II collagen expressing condensation, with the incus and malleus dividing into two due to the upregulation of joint markers, creating two distinct cartilages, in a similar manner to the situation observed in the chick (Amin and Tucker, 2006; Amin et al., 2007). In the mouse this occurs at E14.5, while the incus and malleus do not fully separate until after birth in some mammals (platypus, echidna, opossum) (Anthwal et al., 2020).

The article "Diverse Fate of an Enigmatic Structure: 200 Years of Meckel’s Cartilage" was published in 2020. Journal: Front Cell Dev Biol.

Fossil evidence indicates that Mesozoic mammal-like reptiles had a persistent ossified MCs (Meng et al., 2003, 2011; Luo, 2011; Luo et al., 2015; Anthwal et al., 2017; Mao et al., 2020). Ossification of Meckel’s in these extinct mammaliforms is likely to have provided a support for the malleus and incus as they became integrated in the middle ear while still being physically attached to the mandibular apparatus (Luo, 2011). The loss of the proximal part of MC during mammal evolution allowed for the complete detachment of the middle ear and mandibular units, resulting in enhanced function of the middle ear ossicles, which would then have been able to freely vibrate (Luo, 2011). Loss of MC, therefore, played a key part in the separation of the ear bones from the jaw during the transition from reptiles to mammals (Anthwal et al., 2013).

## Early Development of Mammalian Meckel’s Cartilage

The mandible forms from the first pharyngeal arch and is specified early in development by an absence of Hox gene expression (Hunt et al., 1991). MC forms from within the mandibular mesenchyme, and grafting experiments have indicated it is primarily derived from cranial neural crest cells in birds (CNCCs)(Le Douarin and Dupin, 1993). From mouse lineage labelling studies using the Wnt1cre driver, not all chondrocytes in MC are labelled (Chai et al., 2000; Ito et al., 2002), however, its unclear whether this is due to a substantial non-crest contribution in the mouse or due to the fact that this Cre appears to have different activity in midbrain and hindbrain crest (Chen et al., 2017). Labelling with Mesp1cre, a mesoderm marker, does not label MC or the malleus (Bildsoe et al., 2013). MC has been proposed to be pre-patterned very early on in jaw development, around embryonic day (E) 10 in mice (Ramaesh and Bard, 2003), and initally condenses in the region of the first molar tooth germ at around E11 (Frommer and Margolies, 1971). MC then proceeds to extend anteriorly and posteriorly from this site of initiation (Chai et al., 2000). Formation of MC during mouse development is summarised in Table 1. In human development, condensing mesenchyme cells in the mandible are evident from 32 days (stage 13), with muscular attachments associated with MC observed at 44 days (stage 18) (Wyganowska and Przystanska, 2011). In mice the two rods of MC fuse to create a rostral process (Figure 1B), while in humans the two rods come in close contact but do not appear to fuse (Rodriguez-Vazquez et al., 1997).

**TABLE 1:** Time schedule of MC development in the mouse (as themost common model of MC investigation).

	What happens	How it looks like	References
E8	migration of CNCCs into the 1^st^ pharyngeal arch	undifferentiated ecto-mesenchyme	Chai et al., 1998
E10	clonal expansion of CNCs	undifferentiated ecto-mesenchyme	Takahashi et al., 2001
E11-12	chondroblastic commitment/differentiation	primordium of condensed ecto-mesenchyme	Frommer and Margolies, 1971
E13	chondroblastic differentiation and proliferation, anterio-posterior elongation, fusion of two cartilaginous barsanteriorly	V-shaped structure consisting ofchondroblasts and fibrous tissue, formation of malleal-incudo part posteriorly	Frommer and Margolies, 1971 Amin and Tucker, 2006
E14	rapid growth, anterio-posterior elongation	MC consists of chondroblasts and perichondrium	Sakakura et al., 2007 Ricks et al., 2002
E15	initial hypertrophy of chondrocytes attracts angiogenic cells and precursors of osteoclasts	pre-hypertrophic chondrocytes in intermediate part, TRAP-positive cells apparent on lateral side of intermediate part of MC, malleus separated from incus	Frommer and Margolies, 1971 Sakakura et al., 2005 Amin and Tucker, 2006 Sakakura et al., 2007
E16	binding of Ca^2+^ in hypertrophic region, MC degradation by TRAP-positive cells starts near to mental foramen, blood capillaries penetrate into MC	calcified MC matrix in the intermediate part, TRAP-positive cells and apoptotic bodies cumulate in the area of degradation (apoptotic bodies present also in perichondrium with low frequency)	Ishizeki et al., 1999 Ramaesh and Bard, 2003 Amano et al., 2010
E17	intermediate part of MC disappears	ossification is apparent in the lateral part of the cartilage medially to the mandible	Yang et al., 2012
E18	resorbed area is occupied by osteoblasts, TRAP positive cells and blood capillaries	disconnected anterior and posterior ends of MC, persisting hypertrophic chondrocytes in the posterior portion	Ishizeki et al., 1999
P0	degradation of MC culminates, ossification of middle ear ossicles	chondroblastic cells apparent in the rostral area and posterior region with malleus	Amin and Tucker, 2006 Amano et al., 2010 Anthwal et al., 2013
P3	ossification of middle ear ossicles continues	malleus separates from MC	Anthwal et al., 2013

At E13.5, the mouse MC is composed of small, round and densely packed pre-chondroblasts (Figure 2C). Earlier stages (E12 or E11) are characterised by condensed mesenchymal cells lacking secreted cartilage matrix (Figures 2A,B). Upon differentiation, the chondroblasts become more loosely packed (Figures 2D,D_1_) and reside in cartilage lacuna embedded in extracellular matrix, rich in type II collagen (Frommer and Margolies, 1971). Transverselly orientated clones introduce new cells in columns into MC, controlling the diameter of the rod (Kaucka et al., 2017). This transverse addition of cells from the periphery of the cartilage cannot explain the longitudinal extension of MC, which is therefore presumably due to differentiation of chondrogenic mesenchyme on either end of the cartilage, which is then in turn expanded via the transverse proliferation of chondrocytes (Kaucka et al., 2017). Elongation of MC has been proposed to be driven in part by paracrine factors signalling from the vascular network of the mandibular mesenchyme (Wiszniak et al., 2015). Here it appears that insulin growth factor (IGF), secreted by blood vessels, plays a role in directing growth of MC, with loss of IGF from blood vessels leading to a shorter MC and mandible (Marchant et al., 2020).

The article "Diverse Fate of an Enigmatic Structure: 200 Years of Meckel’s Cartilage" was published in 2020. Journal: Front Cell Dev Biol.

**FIGURE 2:** Histological appearance of Meckel’s cartilage during development. Histological sections of mandible stained with trichrome: sirius red (bone), alcian blue (cartilage), haematoxylin (nuclei). Figures show: frontal section of mandible at E11 **(A)**, 12 **(B)**, 13 **(C)**, 14 **(D,D_1_)** and transversal section of mandible at E15 **(E)**, 16 **(F)**, 17 **(G)**, 18 **(H)**, P0 **(I,J)**. * (molar region), ** (incisor). Taken from slides available in Svandova lab.

At E13 the dentary starts to form (Figure 2C), with MC proposed to have a role in initiating and regulating the growth of the primary ossification centre of the mandible (Frommer and Margolies, 1971). The mandibular dentary bone develops around MC and gradually encases the cartilaginous rod as shown in Figures 3A–C (Anthwal et al., 2008). In other mammalian species, such as the marsupial opossum, MC sits within a groove on the medial surface of the mandible bone and is only encased at the rostral most portion (Anthwal et al., 2017). From E15 onwards the different parts of the cartilage undergo divergent fates.

**FIGURE 3:** Disappearance of Meckel’s cartilage during development. Murine skeletal elements stained with alizarin red (bone) and alcian blue (cartilage) at stages: E15 **(A)**, 16 **(B)**, 19 **(C)**, P1 **(D,D_1_)**, P4 **(E,E_1_)**, P7 **(F,F_1_)**. In figures **(D,E,F)** MC has been dissected away from the surrounding tissues, in figures **(D_1_,E_1_,F_1_)** MC remains *in situ* surrounded by the cranial skeletal elements of the ear and jaw. Gonial bone (GB), incus (I), malleus (M), Meckel’s cartilage (MC), tympanic ring (TR). Taken from skeletal preps available in Svandova lab.

## Diverse Fates Within One Cartilage

In mammals, Meckel’s cartilage can be separated into 3 parts according to the fate of each region: anterior/distal, intermediate/central, and posterior/proximal (Figure 1C). The intermediate part is largely surrounded by the forming dentary bone and is further subdivided into anterior and posterior zones (Bhaskar et al., 1953; Ito et al., 2002; Shimo et al., 2004; Figure 1C).

The article "Diverse Fate of an Enigmatic Structure: 200 Years of Meckel’s Cartilage" was published in 2020. Journal: Front Cell Dev Biol.

From E15, the cartilage cells in the intermediate region continue to mature, having acquired a perichondrium, enlarged lacunae, and a thin matrix in the central part of MC. From this point, chondrocytes adjacent to the ossification centres of the mandibular bone show focal hypertrophy, while the rostral process remains less differentiated (Figure 2E). One day later, the process of hypertrophy culminates (Figure 2F), and is accompanied by type X collagen expression in the intermediate region, while expression of ALP (alkaline phosphatase) is detected in the perichondrium, matrix vesicles and hypertrophic chondrocytes of MC (Ishizeki et al., 1999; Shimo et al., 2004). From E16, calcification of the perichondrium and hypertrophic chondrocytes initiates, with subsequent invasion of the calcified matrix by capillaries (Ishizeki et al., 1999). This blood flow provides bone marrow-derived precursors of multinuclear chondroclasts/osteoclasts that can resorb the calcified cartilaginous matrix (Savostin-Asling and Asling, 1975). New osseous islands are evident at E17 (Figure 2G), which express both type I and type II collagens, and Opn (osteopontin), suggesting a potential contribution of MC to the bone of the mandible (Ishizeki et al., 1999).

Degradation of the cartilage matrix starts around the incisors between E15 and 16 in mice (Figures 2F,G), moving posteriorly toward the molar region and beyond but leaving the most rostral cartilage in place (Figures 2I,J, 3A,B). By E19, the more posterior parts of MC are completely disconnected from the most anterior/distal region (Figures 2H, 3C). This rostral part of MC then either undergoes endochondral ossification to form the mandibular symphysis, or remains cartilaginous in a species dependent manner (Bhaskar et al., 1953). In humans, the rostral region remains cartilaginous, forming nodules on the dorsal surface of the symphysis (Rodriguez-Vazquez et al., 1997).

From the perinatal stage, the most posterior part of MC undergoes endochondral ossification (Figures 3D_1_–F_1_) to form the middle ear ossicles – malleus (Figures 3D–F) and incus (Bhaskar et al., 1953; Frommer and Margolies, 1971; Amin and Tucker, 2006). In mice, the cartilage connection between the mandible and middle ear is still apparent at birth (Figure 3D), but is disconnected by a second site of resportion next to the malleus, resulting in seperation of the ear from the jaw by P4 (Figure 3E; Anthwal et al., 2013). At P7, other than the rostral region and ear ossicles, MC is almost entirely degraded, except for a small nodule next to the dentary (Figures 3F, F_1_). The part of MC adjacent to the ossicles, outside of the dentary, is thought to transdifferentiate to become the anterior ligament of the malleus and the sphenomandibular ligament (Anthwal et al., 2013). In this case, it is proposed that the cartilage matrix is removed and the chondrocytes change to a ligamentous fate. This transformation may involve epidermal growth factor (EGF) signalling, as in the absence of EGF *in vitro* no transformation of MC occured (Ishizeki et al., 2001). From posterior to anterior MC therefore has diverse fates: middle ear bones, ligament, subsumed by the dentary, cartilage.

The article "Diverse Fate of an Enigmatic Structure: 200 Years of Meckel’s Cartilage" was published in 2020. Journal: Front Cell Dev Biol.

## The Removal of the Intermediate Domain of Meckel’s Cartilage

The fate of the intermediate part of MC is unclear. The cells of MC are thought either to contribute to the ossification of the mandible bone, or to undergo cell death (Bhaskar et al., 1953; Richman and Diewert, 1988; Harada and Ishizeki, 1998; Rodriguez-Vazquez et al., 1997; Ishizeki et al., 1999). In either scenario, the matrix of MC is first removed. Meckel’s cartilage extracellular matrix is characteristic of hyaline/hypertrophic cartilage, including the presence of components such as type II and X collagens, aggrecan, versican, decorin, and biglycan (Silbermann and von der Mark, 1990; Shimo et al., 2004; Ababneh and Al-Khateeb, 2009; Tsuzurahara et al., 2011), which provide the mechanical characteristics of cartilage (Shibata et al., 2013). During degeneration of Meckel’s cartilage, metalloproteinases (MMP) Mmp2, Mmp9, Mmp13, and Mmp14 have been detected, with crosstalk among them regulating the degradation of the matrix (Sakakura et al., 2007).

Initially Rank/Opg are expressed at the site of resorption (Sakakura et al., 2005). Then blood vessels, as detected by CD31 expression, bring precursors cells to breakdown the cartilage matrix (Figure 4). These include the precursors of TRAP positive clast cells, as well as macrophages that are observed in the MC perichondrium at E16 and might play a role via stimulation of IL-1β secreted by chondrocytes (Tsuzurahara et al., 2011).

**FIGURE 4:** Distribution of factors suspected to be involved in Meckel’s cartilage degradation. Original schematic showing localisation of osteoclasts/osteoclastic precursors (red = TRAP+), endothelial cells (purple = CD31+) and apoptotic cells (blue = TUNEL+) in the mouse at E14, 16 and 18. Based on the published literature (see Harada and Ishizeki, 1998; Sakakura et al., 2005; Yang et al., 2012).

The ossification hypothesis is supported by the apparent calcification of MC, which starts from the perichondrium on the lateral side, with hypertrophy of the chondrocytes and upregulation of type X collagen (Shimo et al., 2004). Transdifferentiation of chondroblasts into osteoblasts/-cytes has previously been identified during endochondral ossification in other skeletal elements (Yang et al., 2014). Importantly, in cell culture experiments, MC chondrocytes have been shown to be able to transdifferentiate into type I collagen, Alp, Ocn (Osteocalcin) or Osx (Osterix) expressing osteogenic cells (Ishizeki et al., 1996, 1999, 2009; Harada and Ishizeki, 1998; Eames et al., 2004; Ishizeki, 2012). However, the evidence for ossification of the main body of MC through transdifferentiation *in vivo* during normal development is currently limited (Ishizeki et al., 1999). Furthermore, there is no evidence of an ossified MC in species, such as the opossum, where the cartilage is not fully encased by the dentary bone (Urban et al., 2017).

The article "Diverse Fate of an Enigmatic Structure: 200 Years of Meckel’s Cartilage" was published in 2020. Journal: Front Cell Dev Biol.

Alternatively MC cells may undergo cell death following degradation of the cartilage matrix. Apoptosis is the most common mechanism of programmed cell death, however, only a few scattered apoptotic cells have been reported in the intermediate part at E16 and E18 (Trichilis and Wroblewski, 1997; Harada and Ishizeki, 1998; Yang et al., 2012) (summarised in Figure 4). Moreover, of those apoptotic cells associated with MC, the majority were located in the perichondrium, where apoptosis may be acting to prevent the lateral growth of MC (Amano et al., 2010). In agreement with these low levels of apoptosis, the heat shock protein (HSP) 25 is strongly expressed in MC in hypertrophic, proliferative and resting cells and is suggested to protect cells from apoptotic death. Interestingly, down-regulation of Hsp25 results in hypoplasia of the anterior and intermediate parts of MC (Shimada et al., 2003). If apoptosis is not responsible for removal of cells, then other cell death processes might be involved, including autophagy, which is supported by the presence of major autophagic markers Beclin1 and LC3 in the central part of MC (Yang et al., 2012). Beclin1 and LC3, were immunolocalised mostly in prehypertrophic and hypertrophic regions of MC. However, in addition to their engagement in cell death (Bohensky et al., 2014), autophagy has been identified also as a survival mechanism in MC (Song et al., 2017; Luo et al., 2019). Notably, caspase-2 and -8 were found to be activated in the Beclin1 positive regions suggesting a role of these two regulators in autophagy (Bilikova et al., 2019) and indicating that these pro-apoptotic caspases may be acting in a non-canonical manner in MC.

In addition to the intermediate zone, MC also breaks down next to the malleus, separating the ear and the jaw. Like the initial breakdown in the rostal MC, this proximal breakdown point is dependent on chondroclast activity (Anthwal et al., 2017). Interestingly, in the absence of removal of this part of MC by clast cells, in the *cFos* mouse mutant, MC starts to ossify, similar to the situation observed in the mammalian fossil record (Anthwal et al., 2017). Here, ossification appears to be a default state if the cartilage matrix can not be degraded. The loss of Meckel’s cartilage at this point has been recently suggested to be linked to the development of the neighbouring gonial bone, with cartilage cells potentially contributing to the periosteum of this bone (Shibata et al., 2019). No apoptotic cell death has been detected in this region in mice, similar to the situation in the intermediate section, however, there is evidence for apoptosis acting in the disconnection of the middle ear and MC in marsupial opossums (Urban et al., 2017). The exact mechanism for breakdown may therefore be species specific.

The article "Diverse Fate of an Enigmatic Structure: 200 Years of Meckel’s Cartilage" was published in 2020. Journal: Front Cell Dev Biol.

## How Do Meckel’s Cartilage Chondrocytes Compare With Those of Other Cartilages?

There are conflicting opinions as to the characterisation of MC chondroblasts/-cytes when compared to chondrocytes in other cartilages. MC chondroblasts/-cytes are compared most often to those in the growth plate (GP) of the endochondral bone, in particular the limbs. However, mesenchymal precursors of GP and MC chondroblasts are often of different origin, with the cells of MC being mostly derived from the cranial neural crest (CNC), while limb GP cells are derived from mesoderm (Chai et al., 2000). Despite this, several markers, such as Ihh (Indian hedgehog) (Koyama et al., 1996; Nakamura et al., 1997; Shimo et al., 2004), Vegf (Vascular endothelial growth factor) (Carlevaro et al., 2000; Shimo et al., 2004; Zelzer et al., 2004), Sox9, Bmps (Bone morphogenetic proteins) etc. (Mori-Akiyama et al., 2003; Wang et al., 2013; Michigami, 2014) play an important role in differentiation of both MC and GP chondrocytes. Furthermore, metalloproteinases such as Mmp9, 13, and 14, which are known to play important roles in degradation of the extracellular matrix, are found in both endochondral ossification and MC (Vu et al., 1998; Malemud, 2006; Sakakura et al., 2007).

Moreover, MC was found to be affected by a deficiency in trangenic mice of factors known to play a role in GP growth and maturation, including *Fgf3* (Fibroblast growth factor) and Ctgf (Connective tissue growth factor), where proliferation or hypertrophy of MC and GP chondroblasts was disrupted (Shimo et al., 2004).

Molecular signalling proteins do not, however, always have the same distribution and or function in MC and GP cells. For example, Hsp25 (Heat shock protein) is expressed in the GP cartilage in hypertrophic chondrocytes but not in resting and proliferating chondrocytes, however, in MC it was detected from early stage of development in proliferating chondroblasts (Shimada et al., 2003). Specific patterns were observed also for Rankl (Receptor activator of nuclear factor kappa-B ligand), which is expressed exclusively in hypertrophic chondrocytes of GP but is constitutively present in immature and mature MC chondrocytes (Sakakura et al., 2005).

The article "Diverse Fate of an Enigmatic Structure: 200 Years of Meckel’s Cartilage" was published in 2020. Journal: Front Cell Dev Biol.

## The Molecular Biology of Meckel’s Cartilage

The signalling networks within MC are not yet completely understood. Nevertheless, several molecular networks acting in MC patterning, chondroblastic commitment, expansion, differentiation and survival have been identified (Jeong et al., 2004; Liu et al., 2005; Reid et al., 2011; Bonilla-Claudio et al., 2012; Zhang et al., 2013; Billmyre and Klingensmith, 2015) and are summarised here (Figure 5).

**FIGURE 5:** Molecular factors involved in development of Meckel’s cartilage. Original schematic shows key factors identified during formation and disappearance of MC. Factors are clustered according to different developmental events.

### Patterning of the Mandibular Arch

Patterning of the mandibular arch is regulated by several homeobox containing transcription factors including members of the Msx (Msh homeobox), Dlx (Drosophila distal-less), and Tbx (T-box) families. Msx2 is expressed in CNC progenitors, including those that give rise to MC (Davideau et al., 1999). Msx2 was shown to inhibit the chondrogenic differentiation of progenitor cells until CNCCs migration is completed within the mandibular processes (Takahashi et al., 2001). Dlx genes are involved in establishment of the proximo-distal axis in the mandible and maxilla (Depew et al., 2005), coordinated by the Endothelin signalling pathway (Sato et al., 2008; Ruest and Clouthier, 2009). Tbx1 is expressed in the early pharyngeal arch and influences Fgf8 and Bmp4 expression, with its absence resulting in truncated mandible development (Aggarwal et al., 2010). Signalling molecules also play a role in MC patterning. Shh (Sonic hedgehog), although expressed in epithelial domains (Billmyre and Klingensmith, 2015), regulates formation of the mandibular arch derivatives, including MC, as documented in *Shh*-null mice (Melnick et al., 2005). In these mice, increased mesenchymal cell death in the first pharyngeal arch after CNCCs migration was observed resulting in a hypoplastic/missing MC. Formation of the lower jaw and MC also requires endothelin signalling, with a “range of MC defects” in mouse mutants with defects in this pathway (Yanagisawa et al., 1998) (see Table 3).

The article "Diverse Fate of an Enigmatic Structure: 200 Years of Meckel’s Cartilage" was published in 2020. Journal: Front Cell Dev Biol.

### Chondroblastic Commitment and Proliferation

Chondroblastic commitment and proliferation are regulated by secreted factors, including Bmps (Bone morphogenetic proteins) (Denker et al., 1999; Zehentner et al., 1999; Yoon et al., 2005) that appears to be strictly time/site regulated during MC development (Wang et al., 2013). Bmp2 and Bmp7 (but not Bmp4) were expressed in MC at E11.5-12.5 (Wang et al., 2013). Noggin, a negative regulator of Bmp signalling (Zimmerman et al., 1996; Groppe et al., 2002), was expressed in MC during the entire gestation period. In the absence of Noggin, enhanced proliferation was detected with an increased size of MC and a persisting intermediate part (Wang et al., 2013). Proliferation of MC precursors is also regulated by Fgfs (Mina and Havens, 2007; Terao et al., 2011). Fgfr3 is implemented in both, the elongation of MC and the expression of *Sox9* during chondrogenic differentiation (Duplan et al., 2016).

Tgfβ (Transforming growth factor beta) stimulates proliferation of CNC−derived chondrocytes and production of chondroblastic extracellular matrix (Chai et al., 1994; Ito et al., 2002; Oka et al., 2007). Tgfβ signalling acts through intracellular SMADs in a dose−dependent manner, with Smad2 and 3 acting positively, and Smad7 acting negatively (Ito et al., 2002). Tgfβ induces the expression of Ctgf, which is expressed along the entire length of MC (and the perichondrium) from E12.5 to E15.5, playing a role in cell condensation followed by chondroblast differentiation and maturation at later stages (Shimo et al., 2004; Parada et al., 2013). The effect of Ctgf was suggested to result from cell-cell interactions and expression of condensation-associated genes (Ivkovic et al., 2003; Arnott et al., 2011).

### Differentiation and Maturation of Chondroblasts

Differentiation and maturation of chondroblasts is regulated by three master transcription factors Sox9 (SRY-box 9), Runx2 (Runt-related transcription factor 2), and Osx (Osterix) (Zou et al., 2006; Kaback et al., 2008; Nishimura et al., 2012; Zhang et al., 2013). Sox9 (highlighted in Figure 5) is a crucial factor for determination of the chondrogenic lineage in CNCCs population (Mori-Akiyama et al., 2003), promoting the early stage of chondrocyte differentiation (Mori-Akiyama et al., 2003; Yamashita et al., 2009). When *Sox9* was conditionally deleted in CNC-derived cells, differentiation into chondrocytes was blocked, leading to an absence of MC, and instead cells produced osteoblast markers, suggesting their re-specification into an osteoblast lineage (Mori-Akiyama et al., 2003).

The article "Diverse Fate of an Enigmatic Structure: 200 Years of Meckel’s Cartilage" was published in 2020. Journal: Front Cell Dev Biol.

Runx2 is a positive regulator (highlighted in Figure 5) of hypertrophic differentiation (Mikasa et al., 2011; Ding et al., 2012), which acts downstream of IHH (Amano et al., 2014). In MC, Runx2 was found in the zone of hypertrophy (Zhang et al., 2013). *Runx2*-null mice lack all bone and hypertrophic cartilage (Shibata et al., 2004). MC initiates as normal, but has two ectopic cartilaginous processes, which may results from a change in the normal muscle attachment patterns caused by loss of the bone (Shibata et al., 2004). Hypertrophy is also regulated by BMPs (Valcourt et al., 2002; Kobayashi et al., 2005).

Osx plays essential role in osteoblastic differentiation. In MC, Osx was abundantly expressed by hypertrophic chondrocytes and was suggested to be important for conversion of MC chondrocytes into osteoblasts/-cytes (Zhang et al., 2013). In *Osx* null mice, mandibular bone was absent (except for initial condensations), however, the development of Meckel’s cartilage was undistinguishable from the wild type (Nakashima et al., 2002). Since Osx regulates expression of osteoblastic genes, the enhanced expression of osterix in mature chondrocytes might explain the upregulation of type I collagen in these tissues (Nakashima et al., 2002; Zhang et al., 2013). Molecular expression patterns during MC development are detailed in Table 2.

**TABLE 2:** Factors engaged in MC development.

*R (examination at RNA level), P (examination at protein level), A (activity). Patterning of the mandibular arch – grey, proliferation of precursors and chondroblastic commitment – pink, chondroblastic differentiation and hypertrophy – purple, factors of extracellular matrix – green, factors involved in matrix degradation – yellow, factors of cells death – light blue.*

## Consequences of Defects in Meckel’s Cartilage Development

The more posterior parts of the mammalian MC contribute to the formation of two of the three mammalian ear bones (malleus and incus) and associated ligaments (anterior ligament of malleus, sphenomandibular ligament) of the ear and jaw (Ogutcen-Toller, 1995). Defects in the development of these elements lead to hearing loss, as observed in Treacher Collins syndrome and Branchio-oto-renal syndrome (Pron et al., 1993). The very rostral part of MC, remains cartilaginous and contributes to the symphysis. Although a transient structure, the main body of MC supports the development of the mandibular skeleton that forms around it (Ramaesh and Bard, 2003). A number of different mouse mutants that cause reduction or absence of MC consequently develop a shortening of the mandibular bone. For example in *Sox9*^fl/fl^;Wnt1-Cre mouse mutants, the mandibular bones form but are severerly shortened, suggesting that the primary role for the main strut of MC’s is to regulate the length of the mandible (Mori-Akiyama et al., 2003). Other mouse mutants with a reduced MC and shortened mandible include the *Fuz−/−* mice (Zhang et al., 2011) and mice with a first pharyngeal arch deletion of *Shh* (Billmyre and Klingensmith, 2015). Activating mutations in *Fgfr3* lead to abnormal differentiation of chondrocytes and a reduced zone of hypertrophy resulting in shortened skeletal elements, including a truncated MC (Duplan et al., 2016). In this case the activating mutation mimics patients with achondroplasia. A list of transgenic mouse mutants with defects in MC is shown in Table 3.

The article "Diverse Fate of an Enigmatic Structure: 200 Years of Meckel’s Cartilage" was published in 2020. Journal: Front Cell Dev Biol.

**TABLE 3:** Phenotypic abnormalities of Meckel’s cartilageconnected with abnormal gene expression.

Genotype	Impact	References
*Alk2^fl/fl^; Wnt1-Cre* (Bc-MP type I receptor)	missing distal extremity of MC	Dudas et al., 2004
*c-Fos^–/–^*	persistence of MC beyond juvenile stage	Anthwal et al., 2017
*Ctgf^–/–^*	MC deformations	Ivkovic et al., 2003
*Dlx2^–/–^*	abnormal posterior MC, malformed middle ear ossicles	Depew et al., 2005
*Dlx5^–/–^*	MC is shortened and its path back toward the middle ear is disrupted	Depew et al., 2005
*Dlx5/6^–/–^*	complete loss of MC	Robledo et al., 2002
*Dmm/Dmm* (semi-dominant Col2a1 mutation)	growth retardation of MC, osteoarthritis	Ricks et al., 2002
*Ednra constituative activation* *Ednta ^fl/fl^; Wnt1-Cre* *Egfr^–/–^*	transformed upper jaw, with duplication MC duplicated maxilla, loss MC MC deformations	Sato et al., 2008 Ruest and Clouthier, 2009 Miettinen et al., 1999
*Endothelin −/−* *Fgfr3^Y367C/+^*	defect lower jaw, vestigial MC shortened hypertrophic zone of MC, achondroplasia	Ozeki et al., 2004 Duplan et al., 2016
*Fgf8*^neo/^*^–^*	absent or hypoplastic MC	Abu-Issa et al., 2002
*Fuz^–/–^*	hyperplastic malformed MC	Zhang et al., 2011
*Hand 2 ^fl/fl^; Wnt1-Cre* *Isl1^fl/fl^; Shh-Cre*	duplicated mandible and MC smaller MC (E13.5), lack of cartilage at the distal tip resulting in fused growth of two ossifying elements	Funato et al., 2016 Li et al., 2017
*Nog^–/–^*	increased size of MC (due to proliferation) endochondral-like ossification of intermediate part	Wang et al., 2013
*Runx2^–/–^*	two ectopic cartilaginous processes in MC (indirect effect of missing bone)	Shibata et al., 2004
*Setdb1^fl/fl^; Wnt1-Cre*	enlarged MC resulting from increased proliferation and hyperplasia, increased hypertrophy	Yahiro et al., 2017
*Shh^fx^/^–^; Nkx2.5-Cre*	no apparent MC from E14.5	Billmyre and Klingensmith, 2015
*Shh^–/–^*	hypoplastic mesenchymal condensation, no apparent MC	Melnick et al., 2005
*Snai1*^flox/^*^–^ Snai2^–/–^; Wnt1-Cre*	overall shorter length, missing rostral MC and midline fusion	Murray et al., 2007
*Sox9^fl/fl^; Wnt1-Cre*	total absence of MC	Mori-Akiyama et al., 2003
*Sox9 ^+/–^*	MC interrupted and bent toward the body appearing as shortened, campomelic dysplasia	Bi et al., 2001
*Tgfbr2^fl/fl^; Wnt1-Cre* (E14.5)	curvy shape of MC, un-uniform thickness, disrupted perichondrium	Oka et al., 2007
*Tgfβ2 ^–/–^*	abnormal shape of MC	Sanford et al., 1997
*Vegfa^fl/fl^;Wnt1-Cre* (E17.5)	mandibular hypoplasia, decreased size of MC resulting from abnormal vascularisation	Wiszniak et al., 2015

Several human disorders that are directly or indirectly connected with abnormal MC formation have also been described. Similar to the mouse, defects in MC result in the formation of a smaller, malformed dentary bone, resulting in agnathia, micrognathia, or mandibular hypoplasia. Such mandibular defects are fairly common birth defects, with small jaws leading to additional problems associated with airway obstruction and feeding difficulties (Manocha et al., 2019). Mandible defects can be observed in various syndromes including hemifacial microsomia, campomelic dysplasia, Pierre Robin syndrome/sequence, Treacher Collins syndrome, DiGeorge syndrome, and Goldenhar syndrome (Mckenzie, 1958; Bi et al., 2001; Ricks et al., 2002; Wiszniak et al., 2015; Duplan et al., 2016), or be nonsyndromic (see Manocha et al., 2019 for a systematic review). In the case of campomelic dysplasia, causative mutations have been identified in *SOX9*, the master cartilage gene, again highlighing that the microagnathia observed in these patients is due to a defect in MC rather than the later developing dentary (Mansour et al., 2002). In such cases, if the primary jaw defects are due to abnormal development of MC, then the problems could be traced back very early in embryonic development (5–7 weeks), prior to development of the dentary. In the case of Pierre-Robin syndrome/sequence, the formation of a small jaw is thought to have knockon consequences for elevation of the palate, leading to a cleft (Ricks et al., 2002). Similarly, the cleft palate observed in transferrin receptor knockout mice, has been attributed to a failure of Meckel’s cartilage to extend (Lei et al., 2016). As MC contributes both to the jaw and to the middle ear during development, it is perhaps unsuprising that many syndromes, such as Treacher Collins syndrome, combine defects in the jaw and in the ear. In rare cases Meckel’s cartilage fails to breakdown, with the consequence that the jaw and ear remain in physical contact and MC can ossify (Keith, 1910; Herring, 1993). The manifestations of these syndromes are devastating in physical but also psychological aspects and highlight the clinical importance of investigating MC. In addition, understanding the developmental origins of the MC derived anterior malleolar ligament helps to explain why temporomandibular joint (TMJ) trauma can be associated with dislocation of the ear bones (Cheynet et al., 2003). The anatomy only makes sense in the light of an understanding of the development and evolution of the structures.

The article "Diverse Fate of an Enigmatic Structure: 200 Years of Meckel’s Cartilage" was published in 2020. Journal: Front Cell Dev Biol.

## What Is Known and What Remains?

Meckel’s cartilage is an crucial yet transient structure required for the proper formation of the mammalian mandible. The differences in its persistence across jawed animals, and the different fates of the anterior, intermediate, and posterior parts in mammals mean that in understanding the MC we can learn lessons about evolution, skeletal biology, and tissue fate decisions (e.g., Bhaskar et al., 1953; Goret-Nicaise et al., 1984; Ramaesh and Bard, 2003; Amano et al., 2010). Although two hundred years have passed since the discovery of MC, there are still many open questions regarding developmental, cellular and molecular events related to its formation and final fate.

In the mouse model, the timing of the appearance of MC and its propagation and degradation (see Table 1) has been described, the temporospatial pattern of a number genes connected to MC development has been established (see Table 2), and genetic manipulations have pointed to several factors essential for its formation (Sox9, Dlx5/6, Fgf8 or Shh), growth (Alk2, Snail1/2, VegfA) and patterning (Fuz, Noggin, Setdb1) (see Table 3). Both Fgf and Bmp signalling, for example, have been highlighted as involved in non-syndromic lower jaw defects (Manocha et al., 2019).

However, there remain many questions connected with MC. We do not fully understand what induces the formation of MC itself? It is likely that paracrine signals from surrounding tissues play a role, and in line with this a role for Fgf10 has been suggested in early control of MC development (Terao et al., 2011). MC still forms in Fgf10 null mutants (Teshima et al., 2016), however, genetic polymorphisms in Fgf10 have been linked to mandibular prognathism in humans (Cruz et al., 2017). More information is therefore required to understand the identity and location of the signals and how the initiation point for MC is determined. In murine lineage labelling studies the Wnt1cre labelled neural crest cells have been shown to only contribute to a subset of chondrocytes, with the ratios of neural crest and non-neural crest cells changing over time as the cartilage grows (Chai et al., 2000). Whether neural crest cells only form a subset of MC could be tested using a variety of other Cre lines to trace the lineage of cells.

The article "Diverse Fate of an Enigmatic Structure: 200 Years of Meckel’s Cartilage" was published in 2020. Journal: Front Cell Dev Biol.

We also do not fully understand the processes by which MC is removed, in particular the intermediate part. In murine culture, isolated MC persists when dissected out at E14 but degrades when dissected out at E17, suggesting that a cue comes from the surrounding tissue in between these time points (Tsuzurahara et al., 2011). This cue might be molecular or mechanical. For example, it has been suggested that tissue interactions between teeth and MC may induce the breakdown of MC (Sakakura et al., 2005), or that muscle interaction might provide the stimulus for break down (Wyganowska and Przystanska, 2011). A signal might arrive from the surrounding tissue, but equally the signal could be generated from MC itself, stimulating the arrival of macrophages and clast cells to initiate matrix removal (Sakakura et al., 2005, 2007; Tsuzurahara et al., 2011).

Although ample evidence, from *in vitro* studies and mouse mutants, points to MC chondrocytes being able to mineralise (Ishizeki et al., 1999; Anthwal et al., 2017), whether MC ossifies and contributes to the dentary *in vivo* is debated. Novel lineage tracing experiments following the fate of MC cells will be able to address this in future. Such lineage studies would also help to aid our understanding of the transformation of MC into a ligament, shedding light on which cells are involved (perichondrium, chondrocytes) and the nature of the triggers that confine this transformation to just a small subset of the cartilage.

In addition, a number of questions linked to the evolution of MC remain. For example, while the advantage in auditory function gained from removal of the proximal portion of MC during mammal evolution is apparent, the reason for the resorption of the intermediate portion within the mandible is not as obvious. The tapering seen in the ossified MCs of mammal ancestor fossils such as Liaoconodon (Meng et al., 2011) suggests that the anterior MC either degenerated, similar to modern mammals, or may have been present as a cartilage (which did not fossilize). The former might indicate that the resorption of the intermediate MC is more ancient than the breakdown allowing for the separation of the middle ear from the mandible. Interestingly, a late cretaceous mammal has recently been discovered with a tapered ossified MC alongside a decoupled middle ear (Mao et al., 2020). Therefore, perhaps the separation of the middle ear from the MC evolved before the destruction of the intermediate MC. These and other topics remain open and are challenging for further investigations of this transient organ important for evolutionary, clinical and basic research.

The article "Diverse Fate of an Enigmatic Structure: 200 Years of Meckel’s Cartilage" was published in 2020. Journal: Front Cell Dev Biol.

## Concluding Remarks

Here we have charted the evolution, development and clinical aspects of Meckel’s cartilage, highlighting the important role this cartilage plays in the lower jaw. We have detailed the current knowledge but also emphasised the areas where we only have a very basic understanding of the processes involved. With the advent of new lineage tracing techniques, and the availability of conditional mouse mutants, many of these questions are just waiting to be answered.

## Author Contributions

ES wrote the first draft of the manuscript and constructed the figures and tables. NA wrote sections of the manuscript. AT and EM planned the review and finalised the manuscript. All authors contributed to the article and approved the submitted version.

## Conflict of Interest

The authors declare that the research was conducted in the absence of any commercial or financial relationships that could be construed as a potential conflict of interest.
